# Application of Fluorescence In Situ Hybridization Assisted by Fluorescence Microscope in Detection of Her2 Gene in Breast Cancer Patients

**DOI:** 10.1155/2022/3087681

**Published:** 2022-08-11

**Authors:** Fang Lu, Tingting Zhou, Yan Liu, Liying Song, Bin Zhang, Yuyan Li

**Affiliations:** Jilin Kingmed for Clinical Laboratory Co, Ltd., Changchun, Jilin 130000, China

## Abstract

In order to study the important factors for evaluating the prognosis of breast cancer patients, a fluorescence microscopy-assisted fluorescence in situ hybridization technique was proposed. Compared with other detection techniques, fluorescence in situ hybridization (FISH) technology assisted by a fluorescence microscope has gradually gained favor in related fields due to its advantages of high detection specificity, high sensitivity, and strong experimental period. Combined with the basic overview of fluorescence microscopy and FISH technology, the advantages and application points of FISH technology assisted by fluorescence microscopy in the detection of the Her2 gene in breast cancer patients were studied and discussed. The results show that IHC can be used as the primary screening for HER2 gene status detection; IHC (2+) and IHC (3+) have false positives, which are related to chromosome 17 polysomy, so FISH should be done to confirm the diagnosis.

## 1. Introduction

Breast cancer is a common clinical malignant tumor disease in which the proliferation of mammary epithelial cells is out of control under the action of a variety of carcinogenic factors [1]. Data from the Global Burden of Disease Report shows that [2], the age-standardized incidence of breast cancer in women worldwide in 2017 was 45.91 in every 100 thousand people, in the same year, the age-standardized incidence of breast cancer in Chinese women reached 35.62 in every 100 thousand people. The data show that although the incidence of breast cancer in China is lower than the world average, the burden of breast cancer in China has been increasing year by year since 1990, which means that the development of breast cancer prevention and treatment in China will still face great challenges in the future.

Since the publication of human genome research results in 2000, human beings have completed in-depth exploration on the origin of life. In the same year, Perou et al. carried out the first study on breast cancer genotyping, laying an important foundation for future research on the nature of cancer [3]. Human epidermal growth factor receptor 2 (Her2) is one of the breast cancer genes that have been thoroughly studied so far because the overexpression of this gene is closely related to the occurrence and development of tumors [4]. Therefore, in the treatment of breast cancer, the Her2 gene is often regarded not only as an important therapeutic monitoring and prognostic indicator but also as an important clinical target for tumor-targeted therapy [5]. At present, Immunohistochemistry (IHC) and fluorescence in situ hybridization (Fluorescence in situ) are the main techniques recommended by the US Food and Drug Administration for Her2 gene detection. Many studies have confirmed that there are two kinds of hybridization and FISH [6–8]. Although the two detection methods have good consistency in the detection of Her2 gene status, for PATIENTS with IHC (2+), further detection by FISH is more beneficial to obtain more accurate gene status information.

In actual testing work, the FISH will be marked biotin or fluorescein is known sequence specificity of single nucleic acid as a probe, under a certain temperature and ion concentration, with the laws of the complementary base pairing of DNA - DNA in situ hybridization, joint using fluorescence showed that in the end under the assist of fluorescence microscope to determine the DNA in cells to climb biopsy in the original position [9]. In this paper, based on the basic overview of FISH technology and fluorescence microscope, as well as the relevant researches in the recent 20 years, the advantages and application points of FISH technology assisted by fluorescence microscope in the detection of Her2 gene in breast cancer patients were discussed.

## 2. Overview of FISH Technology and Fluorescence Microscopy

### 2.1. FISH Technology

The FISH technique is a nonradioactive molecular cell genetic technique, which is a molecular diagnostic technique based on radiogenic in situ hybridization, using fluorescence markers instead of isotope markers. In 1969, Leung et al. independently developed isotope in situ hybridization technology and pioneered FISH technology. Leung et al. further improved the accuracy of gene localization [10]. In 1974, chromosome banding technology was combined with in situ hybridization technology for the first time. In the following year, Manning et al. connected biotin and RNA molecules through cytochrome C, achieving nonradioactive labeling for the first time. Subsequently, Rudkin and Roumam proposed nonisotope in situ hybridization and fluorescin-labeled in situ hybridization based on the indirect immunofluorescence method in 1977 and 1981 respectively. In 1986, Cassidy and Jones et al. confirmed the feasibility of the FISH technique in interphase nuclear detection of chromosome aneuploidy through experimental studies. Since then, relevant studies on interphase cytogenetics have been started [11]. Since the 1990s, FISH technology has been developing continuously. In addition to the transformation from monochromatic metaphase chromosome FISH to pachytene chromosome FISH and then to fiber FISH, the detection sensitivity of this technology has also been significantly improved. In FISH practice, DNA samples need to be denatured first, followed by the addition of a specific fluorescent-labeled probe, which is promoted to mix and hybridize with the denatured sample DNA, and annealed to obtain fluorescent labeled double-stranded DNA. However, the probe signal in the double-stranded DNA can be captured by a fluorescence microscope, thus achieving qualitative and quantitative detection of sample DNA, as shown in Figure 1. Unlike other techniques, FISH has more operational flexibility and does not require the detection of cells in the phase of division. Therefore, it can be used for the detection and confirmation of gene or chromosome status. In addition, FISH technology can also play an important role in the detection of aneuploid microdeletion syndrome gene rearrangement [12].

### 2.2. Fluorescence Microscope

A fluorescence microscope is a scientific instrument used to study the distribution and location of chemical substances absorbed and transported in cells, mainly through ultraviolet radiation to the object to be examined, so that it fluoresces, so as to realize the shape and position of the object to be checked. A fluorescence microscope is also a kind of optical microscope, but because of its different excitation wavelength from an ordinary optical microscope, a fluorescence microscope has great differences from an ordinary optical microscope in structure and application method. On the one hand, the illumination mode of the fluorescence microscope is mainly falling, that is, the light source is projected on the object to be examined through the objective lens. On the other hand, the fluorescence microscope has two special filters in structure. The filter in front of the light source is mainly for the purpose of filtering out visible light, while the filter between the eyepiece and eyepiece is for the function of filtering out the eyes of the user of the ULTRAVIOLET protection device [13]. As shown in Figure 2, fluorescence microscopy imaging usually goes through the following three steps: (1) First, a light source set up by a fluorescence microscope emits intense ultraviolet light, which is filtered out by an excitation filter. (2) Then, the filtered ultraviolet light will concentrate on the object to be tested under the action of the chromatiscope and induce the fluorescent substance on the object to be tested to emit fluorescence. (3) Finally, under the action of emitting filter, the fluorescence emitted by the fluorescent material will prevent the ultraviolet rays that can threaten human health from passing through, and only the induced fluorescence is allowed to pass through. At this time, the detection personnel can look through the eyepiece and determine the shape and position of the object to be checked according to the fluorescence. At present, fluorescence microscopy is the most widely used method in FISH detection and plays an outstanding role in the qualitative and quantitative study of intracellular substances.

## 3. The Basic Process and Experimental Key Points of the FISH Technique in the Detection of Her2 Gene in Breast Cancer Patients

### 3.1. Advantages of FISH Technology in Detection of Her2 Gene in Breast Cancer Patients

As a nonradioactive detection system, the advantages of FISH technology are mainly reflected in the following aspects: (1) At present, most of the fluorescent dyes and probes used in FISH technology are cheap, and the toxicity of fluorescent dyes is relatively low, which basically does not cause a great impact on living cells, and the safety is good. (2) The probe has high stability and can be used continuously for 2 years after only one labeling. (3) Compared with other detection methods, THE experiment period of FISH technology is short, and the results can be obtained quickly without losing the specificity and accuracy of detection results. (4) The FISH technique is capable of locating DNA sequences up to 1 KB long with sensitivity comparable to that of a radioactive probe. (5) Polychromatic FISH can display many different colors in the same nucleus, so it can realize the simultaneous detection of multiple DNA sequences. (6) The FISH technique has extremely high detection flexibility. The changes in metaphase chromosome number or structure can be detected not only on the slide but also the structure of interphase chromosome DNA can be observed in suspension [14]. Her2 gene is a protooncogene located on the long arm (17Q21) of human chromosome 17 and is an important family member of the growth factor receptor. In recent years, the detection efficiency and quality of FISH technology have improved year by year, and its sensitivity is high [15]. The excellent stability and repeatability of DNA detection, as well as the characteristics of the Her2 gene amplification signal, can still be clearly displayed under the fluorescence microscope oil scope 100 times so that it has become the gold standard to detect whether the receptor pathway of epithelial growth factor cell proliferation and signal transduction is overactivated.

### 3.2. The Basic Process of FISH Technology in the Detection of Her2 Gene in Breast Cancer Patients

In terms of practical application, this paper takes Gajaria and other experimental studies as examples to briefly describe the basic process of FISH technology for detecting the Her2 gene in breast cancer patients [16]: (1) Reagent selection: HemO-DE solvent (xylene substitute), sodium sulfite acid, protease K, washing buffer (2X SSC), wash buffer after hybridization (2X SSC/0.3% NP-40), 0.2 N hydrochloric acid solution, ethyl alcohol of 70/85/100 g/dl, breast cancer Her2 gene test kit (Her2neu DNA probe and CEP17 probe premixed and predenaturated with hybridization buffer). (2) Pretreatment: (i) At room temperature, the tissue sections were immersed in hemo-DE solvent for dewaxing twice, 10 min each time, then immersed in 100 g/dl ethanol for 5 min, repeated twice, and dried; (ii) Under 50°C conditions, tissue sections were treated with 30 g/dl acidic sodium sulfite for 20 min. Then it was rinsed twice with nucleic acid hybridization rinse solution, 5 min each time. (iii) The rinsed tissue sections were immersed in the working solution of protease K and incubated for 20 min under 37 conditions. Then they were rinsed twice for 5 min each time; (iv) After rinsing again, the tissue sections were soaked for 5 min with 0.1 mol/L hydrochloric acid solution at room temperature. After rinsing two times, the tissue sections were placed in −20 precooled 70 g/dl 85 g/dl, 100 g/dl ethanol successively, and dehydrated for two minutes in each row, and then the slides were dried naturally. (3) Probe preparation and sample DNA denaturation: (i) The probe was preheated, the vortex was mixed evenly, and then the transient centrifugation was performed. After centrifugation, the test tube containing the mixture of the probe was placed in a water bath and denatured for 5 min under 73 ± 1°C conditions. After removal, the test tube was placed in a water bath of 45∼50°C until hybridization. (ii) The slides were soaked in 72 denaturing solutions for 5 min, and then the slides were placed in 70 g/dl, 85 g/dl, and 100 g/dl ethanol in sequence for 1-min gradient dehydration treatment and drying; (iii) Drop 10 *μ*L of the probe mixture into the hybridization area of the slides, immediately cover the slides, seal the edges with rubber glue and place in a preheated wet box. Hybridization was carried out in 37 sealed wet boxes for 14–18 h. (4) Posthybridization washes: (i) After hybridization wash buffer was added into the Coplin tank, water bath to 72°C; Add 50 g/dl formamide or nucleic acid hybridization rinse solution to 3 beakers (beaker 1), nucleic acid Hybridization Rinse solution (Beaker 2), 0.1 g/dl ethyl phenyl polyethylene glycol or Nucleic acid hybridization Rinse solution (Beaker 3), Preheat the slides in 451 water bath for 30 min. Remove the cover slides immediately after preheating, and place the slides in beakers 1, 2, and 3 in sequence. Shake the slides for 1∼3 s and let stand for 5∼10 min; (ii) Add the posthybridization washing buffer in another koplin cylinder and place it at room temperature; (iii) After the slides were removed, the rubber adhesive was removed and placed in a posthybridization wash buffer at room temperature to detach the cover glass; (iv) The slides were placed in 72 posthybridization washing buffer for 2 min. They were immersed in 70 g/dl ethanol for 3 min at room temperature (v) They were immersed in 70 gd/l ethanol for 3 min at room temperature. (5) Observe: (i) The DAPI stain was removed and redissolved at room temperature. The DAPI stain was centrifuged for 1∼3 s, followed by whirlpool mixing and a brief centrifugation. The treated DAPI stain was then dropped onto the hybridization area of the slides, and the cover slides were immediately covered; (ii) After standing in the dark for 10–20 min, the slides were observed by fluorescence microscope, and the hybridized slides could be stored in −20 dark condition.

### 3.3. Key Points of FISH Technique in Her2 Gene Detection in Breast Cancer Patients

In practice, there may be some differences in the selection of materials, so the following points should be paid attention to when using FISH technology to detect the Her2 gene: (1) Specimen preparation has an important influence on the accuracy of the test results, especially in the selection of colchicine stimulation to obtain metaphase chromosome division images, the stimulation time is too long or too short, may affect the test results. (2) He et al. found in the experiment that when the concentration of protease K was too high, the morphology of the nucleus would be greatly affected, making it unclear; on the contrary, when the concentration of protease K was too low, it would be more difficult for the probe to enter the nucleus, resulting in a lower success rate of hybridization [17]. In terms of paraffin sections, digestion of 20 g/L protease K for 20 min at 50 conditions could maintain the success rate of hybridization at a high level without destroying nuclear morphology. (3) At the present stage, although there are a wide variety of probe kits on the market, big brand kits should be used in the selection, and there are more or fewer differences in the use of enzymes in the kit from different manufacturers, so the experiment should be carried out strictly according to the operation steps and conditions in the instruction manual. (4) Zhan et al. gave suggestions based on the experimental results [18], the optimal hybridization conditions for FISH detection were 37 to 40 overnight in a wet box protected from light, and incubation time was between 18 and 20 h. However, automatic DNA unchain was easy to occur when the incubation time was longer, leading to signal reduction. (5) The FISH experiment is sensitive to temperature, so the temperature of the rinse solution should be raised to 37 rather than room temperature when rinsing. (6) Shah et al. pointed out that the object to be tested should be detected and observed as soon as possible after sealing because each fluorescence microscope observation would quench part of the signal. Therefore, observation and image collection should be completed quickly in the FISH experiment to prolong the service life of the sample [19].

## 4. Advantages of Fluorescence Microscope and Key Points of Application in Detection of Her2 Gene in Breast Cancer Patients

### 4.1. Advantages of Fluorescence Microscopy

Compared with the ordinary light microscope, the fluorescence microscope has the following advantages: (1) High specificity and sensitivity, even under the condition of a very low concentration of fluorescent dye, it can still be detected in the object to be detected with a very low content of the target substance [20]. (2) The sample preparation process is simple and the observation procedure is simple, which is more suitable for the rapid identification of target substances. (3) With the development of various new fluorescent dyes, the range of substances to be measured is also expanding.

### 4.2. Application of Fluorescence Microscopy in Detection of Her2 Gene in Breast Cancer Patients

Fluorescence microscopy also plays an important role in FISH's detection of the Her2 gene in breast cancer patients [21]. Rational use of a fluorescence microscope is not only beneficial to prolong the service life of the instrument but also of great significance to improve the accuracy of detection. Therefore, the following points should be paid special attention to in the practical application of fluorescence microscope [22]:

(1) Preinspection and adjustment is an important step before the use of a fluorescence microscope. Before each fluorescence observation, the inspector should first perform a routine inspection on the filament pair of the fluorescence device, the focal aperture, the aperture, the field of view, and the setting of the aperture; Secondly, inspection personnel should carefully check whether the excitation filter and emission filter components are correctly installed on the converter before use. In addition, they should also confirm whether the objective lens is properly configured and thoroughly remove oil stains and dust on the lens in front of the objective lens with corresponding cleaning utensils [23]; Finally, because the fluorescence microscope takes ULTRAVIOLET light as the main lighting source, and although the transmitting filter can effectively block ultraviolet light, ultraviolet light may be refracted to the object platform, and then cause harm to the human body, therefore, a suitable size of the brown shade should be placed in front and above the object platform before the instrument is used. In addition, a voltage regulator should be installed between the instrument and the power supply to ensure that the voltage stability is maintained at the same level during the life of the instrument since voltage instability will destroy the service life of the high-pressure mercury lamp [24].

(2) After preparing for the test, the power can be turned on, but after the fluorescent lamp source is turned on, it should be left for 5∼10 min until the excitation light intensity is stable, and then the object to be measured is placed on the carrier and observed; In focus or looking for object detection, need through the narrow aperture of the fluorescence illuminator, or take other appropriate method to reduce the intensity of excitation light, to determine the mirror, then raise the excitation light intensity to the best state, by this operation, can effectively avoid the excitation light fluorescence quenching caused by excessive exposure to the sample [25]; In addition, in addition to sample preparation and other related factors, when the image quality is found to be poor, the image quality can be improved one by one by checking, and adjusting the focusing of the receiver of the blocking or light limiting device in the imaging optical path and the objective lens coverage checking and correcting ring of the aperture aperture.

## 5. Conclusion

Through the analysis of this experiment, we believe that immunohistochemistry is easy to carry out in ordinary laboratories, and the results are highly consistent with FISH and can be used as the primary screening for the detection of HER2 gene status; however, due to the influence of various factors, there are False negative or false positive, so when determining the treatment method clinically, the HER2 gene status should be based on the FISH test results. Fluorescence microscopy and FISH technology have extremely high application value in the detection of the Her2 gene in breast cancer patients. Combining the technical advantages of fluorescence microscopy and FISH, according to the development of related technologies, fully grasp the application of fluorescence microscopy-assisted FISH technology in the detection of the Her2 gene in breast cancer patients. To ensure that it plays a greater role in breast cancer prevention and treatment.

## Figures and Tables

**Figure 1:** FISH flow chart.

**Figure 2:** Schematic diagram of fluorescence microscope principle.

## Data Availability

The data used to support the findings of this study are available from the corresponding author upon request.
